This article has been retracted.

# Challenges and Optimization Paths of Guzheng Professional Education in Colleges under Big Data Era

**DOI:** 10.1155/2022/4941860

**Published:** 2022-09-06

**Authors:** Li Cheng, Liang Hu

**Affiliations:** Music College of Yangzhou University, Yangzhou, Jiangsu 225000, China

## Abstract

As a treasure among Chinese national musical instruments, guzheng is an important part of traditional Chinese music. As the art of national music goes to the world, the art of guzheng has been widely promoted. As the best form to carry forward the art of guzheng, the teaching of guzheng majors in colleges is significant in teaching and continuously improves guzheng art accomplishment. Oral teaching and step-by-step music theory and technique teaching are typical ways of teaching musical instrument performance in colleges. However, under big data, Chinese education is undergoing a profound change, and the combination of big data and education has become a new contemporary education method. This work studies the guzheng professional education in colleges under big data. First, this work aims at the existing outstanding issues of guzheng teaching in colleges and studies the challenges and optimization paths of guzheng professional education in colleges under big data. Second, this work proposes a multiscale residual attention fusion network (MSRAFNET) to evaluate the teaching quality of guzheng majors in colleges in the era of big data. The feature extraction of the network model is mainly completed by the residual module, which is composed of several multiscale residual learning units. Adding an attention mechanism to the multiscale residual learning unit can enhance the feature extraction of key information by the network and reduce the interference of redundant information, which is more conducive to the learning of data features. It adopts the design of GAP and Dropout to reduce spatial parameters in network training, and the effect of antioverfitting is better. Third, this work systematically evaluates the optimization path of Guzheng education and MSRAFNET, and the systematic experiments verify the superiority of the designed method.

## 1. Introduction

Ancient Chinese musical instruments have a history of thousands of years of development, and, among them, the guzheng has become a national treasure recognized by people. With continuous development for society, the guzheng has become a musical instrument that is appreciated by both refined and popular people. The art of guzheng has developed rapidly in recent decades. From the creation of guzheng music to the increase in the number of people learning guzheng from professional to amateur, we can see the development of the traditional guzheng industry. At the same time, with the continuous improvement of comprehensive national strength, the guzheng has stepped onto the big stage of world development. However, in the actual guzheng teaching, there are still various problems and deficiencies, which need to be paid attention to by colleges. Under this background, the guzheng majors in colleges should choose suitable methods to carry out teaching and cultivate students' interest in learning, and students can be more active in classroom knowledge learning and improve their own guzheng knowledge and skills. More and more students who love traditional culture and art take the guzheng elective study, which not only brings an opportunity for the dissemination of excellent classical music and art and the promotion of traditional culture but also makes the traditional guzheng teaching methods and teacher resources in colleges show insufficiency. Whether these problems can be solved via big data, better dissemination of guzheng music art as well as the exploration of its excellent national culture and ideological value is a topic worth exploring [1–7].

Each stage of guzheng learning is based on the science of playing technique and physiology, and each stage of learning has different styles and genres of repertoire. This requires students to thoroughly understand the works, correctly grasp the content and characteristics of the works, and improve performance skills in process of learning the guzheng. The purpose of guzheng teaching in colleges is to train and educate students, and guzheng teaching is also opened and increased year by year. First of all, the teaching of guzheng can cultivate students' moral sentiments, and, through the teaching of guzheng knowledge, music can be used to develop students' intellectual potential. Guzheng is a treasure of Chinese traditional culture and traditional art, which contains profound cultural heritage. It can express multilevel and profound connotations through contagious music, adhering to the development concept of the unity of guzheng people or learning from nature, and can subtly nurture and cultivate students' noble moral sentiments. This enables students to experience the profound cultural connotation of guzheng and improve their self-cultivation. Secondly, guzheng teaching can improve students' own artistic accomplishment. The so-called artistic accomplishment is a kind of cultivation of students' own inner aesthetic ability and appreciation ability. The teaching of guzheng knowledge needs to be gradually accumulated before it can be carried out. Guzheng is a treasure of ancient Chinese national art and culture. It has the characteristics of classical elegance and can cultivate students' own traditional cultural heritage. When teaching guzheng knowledge, teachers can cultivate students' interest in learning through the beautiful and pleasant music played by guzheng strings, create a harmonious classroom learning atmosphere, and enable students to deeply feel the beauty of guzheng music [8–14].

At present, the scale of guzheng professional education is improved in stages. In recent years, learning Guzheng has been loved by music lovers at home and abroad and is very popular among students in colleges. In addition to major music colleges across the country, many nonart colleges have also opened guzheng majors. The gradual deepening of guzheng majors in ordinary colleges is conducive to strengthening the theoretical research on guzheng instruments and the inheritance and development of guzheng art. The playing technique of guzheng has also been developed by a breakthrough. The original playing method of guzheng is to play the melody with the right hand. It adjusts the change of string sound by pressing, sliding, kneading, chant, and other techniques, so as to beautify the tone and express the style characteristics. By the end of the twentieth century, the playing technique of guzheng had achieved a breakthrough development, and the technique of polyphony was used in the tune, which greatly enriched the playing skills. This kind of application from playing with one hand to playing with both hands and then from the appearance of the remote thumbwheel finger to the application of fast fingering sequence makes the guzheng more attractive and deeply loved by people. In addition, guzheng creation is influenced by western composition. In process of guzheng major education in colleges, it has been deeply influenced by western composition skills and aesthetic viewpoints, that is, listening habits. The content of Chinese guzheng creation has also changed, and many new music works have been created, which has injected fresh blood into the teaching of guzheng [15–20].

This work studies the guzheng professional education in colleges under big data. First, this work aims at existing outstanding issues of guzheng teaching in colleges and studies the challenges and optimization paths of guzheng professional education in colleges under big data. Second, this work proposes a MSRAFNET to evaluate the teaching quality of guzheng majors in colleges under big data. The feature extraction of the network model is mainly completed by the residual module, which is composed of several multiscale residual learning units. Adding an attention mechanism to the multiscale residual learning unit can enhance the feature extraction of key information by the network and reduce the interference of redundant information, which is more conducive to the learning of data features. It adopts the design of GAP and Dropout to reduce spatial parameters in network training, and the effect of antioverfitting is better. Third, this work systematically evaluates the optimization path of Guzheng education and MSRAFNET, and the systematic experiments verify the feasibility and superiority of the designed method.

## 2. Related Work

Literature [21] found that the goals and reasons for students to participate in guzheng learning were not clear enough. Many students followed the plans set by their classmates or their parents to participate in guzheng learning. Students had many misunderstandings in the process of guzheng learning. Teachers did not have a very standardized and scientific teaching plan for guzheng teaching. In their usual teaching, they mainly focused on guzheng music performance, and the teaching of music theory was not enough. Most of the guzheng teaching did not have uniform and standardized teaching materials. In response to these problems, the author put forward some countermeasures to solve the problems. Literature [22] analyzed the current situation of social guzheng teaching. At present, the level of institutions in social teaching is uneven. The selection of teachers was not strictly checked, and the selection of teaching materials and teaching methods could not pay attention to cultivation of abilities. Therefore, effective measures were proposed. Literature [23] introduced the current situation of teachers' quality in teaching. At present, there are several problems of low teaching ability, low professional ethics, and low professional level of guzheng teachers, and some suggestions were put forward for these problems. Literature [24] found that 80% of students did not have lasting interest in learning, and it was proposed that cultivating interest was an important factor in learning the guzheng well. Teachers should play a guiding role, focused on cultivating students' interests in teaching, and teach students in accordance with their aptitude. Reference [25] made a detailed analysis of the musical structure of the work. The paper talked about the harmony setting, melody trend, and artistic expression from the musical structure analysis of the piece. Literature [26] discussed the notation characteristics, mode characteristics, variation characteristics, plate characteristics, rhythm characteristics, and technical characteristics of guzheng music. This paper provided a lot of theoretical reference for the music analysis of guzheng music. The author of [27] made a detailed study on the creative techniques of traditional guzheng music, including the development of melody, the modulation of guzheng tune, the polyphony of guzheng tune, and the musical structure of guzheng tune. His thesis also discussed the influence of the creation of traditional guzheng music on modern guzheng tunes and analyzed some modern guzheng tunes that were more characteristic in their creation techniques.

Literature [28] divided the perception of music into outer, middle, and inner layers. The outer layer was only the understanding of the musical score, and, in order to achieve the middle layer of music perception, it was necessary to analyze and understand the music and then comprehended the character, charm, and spirit of the music, which was the inner layer of music perception. The application of music analysis to guzheng teaching was to improve students' aesthetic ability from the inner music perception. Literature [29] believed that the teaching of guzheng should be a comprehensive teaching, which should be carried out comprehensively and deeply in combination with the practice of language movements and performances. Literature [30] pointed out that the current guzheng teaching was too simple and proposed the Guzheng teaching method of theoretical guidance. In the guzheng class, teachers first let students learn the knowledge of music theory and then carried out technical practice. Literature [31] mainly adopted the research method combining case study method, interview method, and direct observation method and took the guzheng training center as the main research position. It refined the teaching concept of the Guzheng basic teaching method, excavated the advantages and theoretical basis of the Guzheng basic teaching method, and drew a conclusion that the Guzheng basic teaching method was worth popularizing in the primary stage of the Guzheng basic teaching. Literature [32] discussed the application of excellent teaching methods in guzheng teaching. It also enumerated the specific teaching cases of these teaching methods used in the teaching of Guzheng. Reference [33], based on its own teaching practice experience, researched a set of teaching methods of group class composite mode that was more in line with actual needs. By organically combining the group and the individual in the group class, it could not only ensure the full play of the advantages of the group class but also ensure the effect of one-to-one teaching as much as possible. Literature [34] conducted an investigation and interview with teachers and students by taking the collective teaching of guzheng in the second classroom activity as a practical exploration point. It summarized and analyzed the resistance to the development of the Guzheng collective class teaching mode at the current stage and the problems existing in the teaching process. It took two semesters to carry out teaching practice in the school, and a set of practical and effective teaching methods and models that could be applied to guzheng group classes were gradually formed. Literature [35] introduced the traditional teaching and MOOC teaching mode of Guzheng and, on this basis, listed the advantages and disadvantages of the two teaching modes through the method of comparative research. It tried to integrate the two teaching modes, so as to find a more scientific and advanced Guzheng teaching mode.

## 3. Method

This work studies the guzheng professional education in colleges under big data. First, this work aims at existing outstanding issues of guzheng teaching in colleges and studies the challenges and optimization paths of guzheng professional education in colleges under big data. Second, this work proposes a MSRAFNET to evaluate the teaching quality of guzheng majors in colleges under big data. The feature extraction of the network model is mainly completed by the residual module, which is composed of several multiscale residual learning units. Adding an attention mechanism to the multiscale residual learning unit can enhance the feature extraction of key information by the network and reduce the interference of redundant information, which is more conducive to the learning of data features. It adopts the design of GAP and Dropout to reduce spatial parameters in network training, and the effect of antioverfitting is better.

### 3.1. Challenges and Optimization Paths of Guzheng Professional Education

More and more students are enrolled in the guzheng major courses in colleges, which makes the inheritance of the ancient musical instrument performance skills and works creation show an unprecedented prosperity. However, some problems and contradictions in the teaching of guzheng are also more obvious.

First, there is a relative shortage of teachers specializing in guzheng teaching in colleges. Although, under big data, people have come into contact with a variety of music arts and cultures, the inheritance of national music was initially affected to a certain extent, and the general audience was divided by popular music with changing styles all over the world. But, on the other hand, by learning more types of traditional and modern music, more younger generations have realized the value of traditional folk music art. In particular, the performance of national musical instruments represented by the guzheng, as an important element in the spiritual and cultural life of generations of ancestors, attracts more and more college students to study and also makes the ratio of guzheng teachers and students in colleges tend to be unbalanced. The improvement of guzheng playing skills is very dependent on teachers' one-to-one guidance and intuitive demonstration teaching.

Second, existing guzheng teaching mode cannot meet learning needs of students under big data. At present, most of students' guzheng-related courses in colleges are elective courses, not the first major. Therefore, most of the students hope to master the performance skills of this traditional national musical instrument in the study of music majors and enrich their national artistic accomplishment. However, the guzheng teaching in colleges does not make arrangements for the different learning needs of students but sets up courses according to the traditional systematic teaching mode of guzheng majors. It starts with the most basic relevant theoretical knowledge and then gradually explains various traditional and modern playing techniques and styles. This teaching mode not only fails to meet the expectations of nonguzheng majors to learn to play the guzheng as soon as possible but also has its inappropriateness for the guzheng majors. This is because, under big data, college students are more eager to maintain a personalized artistic style and have a unique understanding of musical instruments and musical works. Therefore, in the process of learning guzheng, we hope to get more equal exchanges and hope to have the opportunity to show the progress and inspiration of music and art made by individuals in the process of learning guzheng. The existing teaching models cannot meet these.

Third, colleges focus too much on music theory and performance skills and ignore the dissemination of cultural and artistic connotations. The traditional guzheng teaching methods and course content structure have a large proportion of basic theories, and this theoretical knowledge is very necessary for students majoring in guzheng. However, under big data, students who choose to learn to play guzheng are not only inspired by the artistic charm of this classical national musical instrument and its musical works. A large part of the reason is based on admiration for traditional culture and artistic ideas, hoping to improve personal cultural and artistic accomplishment by learning guzheng and experience the spiritual world enriched by the ancients by qin, chess, calligraphy, and painting. Therefore, guzheng teaching in colleges only regards the guzheng as a musical instrument and regards guzheng teaching simply as teaching the playing skills of a musical instrument, lacking the comprehensive inheritance of related traditional culture and art. Therefore, on the one hand, they did not make good use of students' enthusiasm for learning to inherit the excellent national culture and missed the rare opportunity to carry forward traditional culture in the Internet age. On the other hand, students' learning will not get the expected results.

Aiming at the existing issues, this paper explores the use of the new interactive mode and abundant resource advantages brought by big data to find feasible measures to solve these problems.

First is changing teaching methods according to the individual needs of contemporary students. Guzheng teaching in the era of big data should be based on students' individual learning needs, provide a relatively relaxed learning environment, and give students more choices in course content. Therefore, by refining the classification of guzheng teaching courses, different curriculum systems can be provided for students who major in guzheng majors and electives. Therefore, on the premise of ensuring that students majoring in guzheng have a solid theoretical foundation, students who elect to take guzheng can choose specific content based on their personal learning goals.

Second is building a guzheng teaching and communication platform based on big data. Under big data, college students are willing to display themselves and obtain required information on the network platform. Teaching in many disciplines has been remote teaching through online platforms or providing students with learning resources. Students who learn guzheng do so basically out of personal love for traditional music art and related culture. Therefore, they not only have a strong desire to communicate and interact but also urgently need a platform to display the results of their personal learning of guzheng. Therefore, in view of the relative shortage of teachers in guzheng teaching in colleges and the inability to provide students with enough practical opportunities, we can build a guzheng network teaching platform.

Third is excavating network teaching resources to spread the music art and cultural thoughts related to guzheng. The reason why guzheng has shown great charm to college students under big data is that it is inextricably linked with traditional Chinese culture. The purpose of students learning guzheng is not only to obtain a certain level of performance skills but also to hope that, through learning guzheng performance, they will reach a higher level in terms of personal culture and artistic accomplishment. Therefore, teachers should tap the rich teaching resources on the Internet, on the one hand, to meet the students' deeper learning needs and, on the other hand, take the opportunity to spread the music, art, and cultural ideas related to the guzheng and seize this opportunity to inherit China's excellent cultural and artistic heritage.

### 3.2. CNN Knowledge

CNN generally inputs sample data in input layer, uses hidden layer to learn information, and reduces dimensionality of a large amount of data in training and finally uses the classification function to identify and classify the data. When the CNN is trained, the backpropagation algorithm calculates the error, and the network uses the error to update each parameter to achieve purpose for correct identification. It is necessary to utilize local perception and weight sharing, which are also the two major characteristics of CNN networks.

CNN's most critical component is the convolutional layer. This layer is mostly used to perform convolution operations on data from the input layer in order to extract features. To further process the data entered into the convolution layer, one or more convolution kernels are utilized, with each convolution kernel serving as a filter. For each convolution kernel, the parameter values will vary and so will the features that are extracted from the input data. The number of network parameters can be considerably decreased by setting a sensible convolution kernel size such that each neuron is only connected to a local portion of the feature map output by the preceding convolution layer. It is the number of pixels that the kernel moves in the width and height directions of the feature map each time. The smaller the feature map generated by the convolution operation, the larger the convolution step size. Before the convolution procedure, the feature map's boundary is intentionally zero-padded, allowing the convolution kernel to be calculated beyond the original feature map's boundaries. Because of this, the size of the feature map produced by a convolution operation depends on three variables: the kernel, stride, and edge padding.

(1) $$\begin{array}{c} h_{c}=\frac{\left(h_{i}-h_{k}+2\text{pad}\right)}{s_{h}}+1,\\ w_{c}=\frac{\left(w_{i}-w_{k}+2\text{pad}\right)}{s_{w}}+1, \end{array}$$

where *h*_*i*_ and *w*_*i*_ are the sizes of input, *h*_*k*_ and *w*_*k*_ are the sizes of kernel, and *s*_*h*_ and *s*_*w*_ are the step sizes.

The pooling layer is to imitate the human visual system to perform downsampling operations on a large number of feature maps obtained after convolution operations. It discards redundant features while retaining important features to achieve dimensionality reduction for feature maps. The pooling operation can make the feature map smaller, but it does not change the number of feature maps. Max pooling is utilized to extract the local maximum value, and average pooling is utilized to extract local average value in the feature map. Pooling layers have no parameters that need to be updated during training, so adding pooling layers to a convolutional neural network does not increase parameters. The calculation rules are

(2) $$\begin{array}{c} P_{\text{max}}=\underset{0<i,j<K}{\max}x_{ij},\\ P_{\text{avg}}=\frac{1}{K\times K}\sum_{i=1}^{K}\sum_{j=1}^{K}x_{ij}, \end{array}$$

where *x*_*ij*_ is feature.

In the neural network, the convolution and pooling operations are all simple linear operations. A large number of linear operations seriously affect the extraction of feature information by the network model, making the network unable to deal with complex problems. The activation function can improve the problems caused by a large number of linear calculations in the model and improve ability to extract feature information.

Fully connected layers have every neuron linked to every neuron in the prior layer. The fully connected layer's job is to bring together the deep features that have been retrieved through a series of convolution and pooling processes. Fully connected layers are usually responsible for most of the parameters in convolutional neural networks. Increasing parameters in the fully connected layer can increase the model's complexity, which in theory can improve the model's learning ability. However, if the number of fully linked layer parameters is too great, the model will take longer to run and be more susceptible to overfitting. To ensure that the convolutional neural network performs better, it is vital to limit the number of parameters of the fully connected layer in the experiment. The calculation is

(3) $$\begin{array}{c} y=f\left(\sum_{i}w_{i}x_{i}\right), \end{array}$$

where *w*_*i*_ is weight and *x*_*i*_ is feature.

The output layer's primary function is to sort the input data into several categories. Convolutional neural networks commonly use Softmax classifiers to categorize one-dimensional feature vectors that are output by the fully connected layer in multiclassification tasks. If the input data is classified as belonging to more than one of several categories, the classifier's final outcome will be the category with the highest probability, and the probabilities for each category's total are guaranteed to be one.

During the training process of convolutional neural network, it is easy to occur that the convolutional neural network performs well on training set but performs generally on validation set and test set. This means that the convolutional neural network model has poor predictive ability for unknowns and generalization ability; that is, overfitting occurs. The Dropout method is to alleviate the occurrence of overfitting by modifying CNN. During training process of convolutional neural network, the Dropout method randomly stops some neurons from working with a certain probability, and the neurons that stop working do not update the weights of the neurons in the current iterative training.

According to machine learning, training and testing data must both have the same probability density. Convolutional neural networks have to learn a new distribution for each iteration of training, since the distribution of each batch of training data differs somewhat in practice. As a result, the network model faces difficulty in learning the input data distribution law consistently, which significantly slows down the network's training time. A convolutional neural network's input data is normalized in batches using the batch normalization (BN) method, which yields data with a standard normal distribution that can be used as input for training. It is possible that, after BN processing, the majority of the activation function values will fall inside the linear range. It allows network models to have strong nonlinear expression abilities and to avoid the problem of slow network convergence due to the loss of gradients.

### 3.3. MSRAFNET Algorithm

This work proposes a MSRAFNET framework for evaluating the education quality of guzheng majors in colleges under big data, and its structure is demonstrated in Figure 1.

This work proposes a multiscale residual learning (MSRL) unit, which includes three branches. Two are branches containing convolutional layers, and the remaining one is an identity mapping branch. The branch including the convolution layer uses a small convolution kernel and sets different numbers of convolutions to extract different features. The structure is demonstrated in Figure 2.

The multiscale residual learning unit utilizes two branches containing convolutional layers to perform multiscale feature extraction. The first 1 × 1 convolution of each branch reduces the dimensionality of the input so that the dimensionality of the 3 × 3 convolution is not affected by the network. If the convolution numbers of the two branches are different, the features extracted by the two branches are different. The differently extracted features are fused using the concat method, which combines the channel numbers of the two feature maps that need to be fused to achieve the purpose. The fused features are dimensionally increased by 1 × 1 convolution to ensure that the dimensions of the input and output are equal, so that more abundant features will be obtained to improve the accuracy.

The multiscale residual learning unit can perform multiscale feature extraction on the input data but cannot extract the information of the adjustment key local area. Therefore, this work combines it with an attention mechanism to propose a multiscale attention residual (MSARL) learning unit. The attention mechanism redistributes and weighs the weights during network training. The key local area of the feature needs to be focused on learning and the weight is set to be large, and the noncritical area only needs to be assisted by learning, so the weight is set to be small, so that the key information of the feature can be extracted.

Spatial attention mechanisms, channel attention mechanisms, and hybrid attention mechanisms are the most common strategies for focusing attention. Focusing on the spatial realm is what the spatial attention mechanism does. To begin, the input feature map is averaged and maximized to produce the final feature map. To obtain the feature map, do a convolution and then apply the sigmoid activation function. The extracted spatial information from the feature map is obtained by multiplying the input by the attention mechanism's weights, and the ultimate output is a feature map. The calculation is

(4) $$\begin{array}{c} Att\left(sp\right)=\text{sigmoid}\left(f_{\text{conv}}\left(f_{\text{concat}}\left(f_{\max}\left(x\right)+f_{\text{avg}}\left(x\right)\right)\right)\right), \end{array}$$

where *f*_conv_ is convolution operation and *f*_concat_ is concat operation.

Channel attention will focus on feature map channel information and process it. The weighting operation is performed on channel, the key area is given a large weight, and the feature extraction of this part is strengthened to ignore the nonkey features. This is more conducive to extracting the important information of the image and improving the network performance. This method realizes the function through the compression module and the excitation module.

(5) $$\begin{array}{c} Att\left(ch\right)=F_{\text{scale}}\left(u_{c},s_{c}\right), \end{array}$$

where *u*_*c*_ and *s*_*c*_ are feature operations.

This work combines spatial attention with channel attention and uses a hybrid attention mechanism to build a multiscale residual attention learning unit, as demonstrated in Figure 3.

This module uses two branches with different numbers of convolutional layers to extract multiscale features. It extracts features of the expression data through these two branches and uses the concat method to fuse the features. The fused features are processed by a hybrid attention mechanism, which enables the network to assign greater weight to key regions and learn more important features.

With deepening of network, parameters involved in the operation will continue to increase, and a large amount of redundant information will also be generated. If these parameters are not processed, the speed of network training will become slow, and it will easily lead to overfitting problems and reduce the recognition rate. This work proposes a transition layer structure, as demonstrated in Figure 4.

The transition layer consists of a 3 × 3 convolution and Max pool. 3 × 3 convolution increases the dimension when extracting features, increases the linear transformation capability of the network, and increases the dimension of the input to the next residual module. Max pool performs downsampling operations, which can reduce the size of the parameter matrix, and Max pool can adapt to pixel translation and rotation operations. Therefore, the maximum pooling is used to reduce interference information, parameters, and calculation.

In CNN, the network is often made more complex by increasing the number of layers of the network, and then the features with strong discriminative power are extracted. In this way, new problems will arise, and the network can more accurately identify the training set data during training. However, when using a trained model for prediction, the high accuracy during training is often not achieved, which is called overfitting. The main reason for overfitting is that the relationship between sample labels and familiar information is overlearned in the training process, and a large amount of interference information is also regarded as the key feature of the data, which leads to a great reduction in the recognition accuracy. The general neural network will choose an FC layer followed by an activation function. However, use of the fully connected layer will lead to a sharp increase in the parameters involved in the training. The network training speed is slow and overfitting is easy to occur. GAP can effectively solve this phenomenon. The fully connected layer uses each vector to correspond to each feature map for classification. GAP adopts the global mean pooling operation and uses the one-to-one correspondence between feature and output for classification, which directly realizes dimensionality reduction. This reduces the amount of computation during training and has a good antioverfitting effect.

Adding Dropout to the network structure will randomly make some neurons no longer participate in training. This makes the exchange of information no longer close, and the network can further learn the internal relationship of the data. Specifically, during the forward propagation of neurons, setting the value of some neurons to zero is equivalent to randomly letting the neurons no longer transmit the output value to the lower layer to participate in the training process. During backpropagation, these neurons also no longer operate. Adding Dropout to the network makes the training results less dependent on some local features and improves the generalization ability of the algorithm.

This work chooses to use GAP and Dropout design. The total amount of guzheng professional education data in colleges is small, and overfitting is easy to appear in the training process. Therefore, this layer needs to be added to ensure the normal progress of the training process.

## 4. Experiment

### 4.1. Evaluation on MSRAFNET

This work collects data related to teaching of guzheng majors in colleges to construct the dataset. The data features contained in each sample are demonstrated in Table 1, which are expanded into 256 × 256 format data to meet requirements of network. The label of each sample is the corresponding guzheng teaching quality. The experiments are based on the PyTorch framework of Python, the hardware configuration is NVIDIA GTX 1080Ti GPU, the video memory is 8 G, and all experiments are completed under the Ubuntu operating platform. The utilized evaluation metrics are precision and recall, and the calculations are as follows:

(6) $$\begin{array}{c} \text{Pre}=\frac{\text{TP}}{\text{TP}+\text{FP}},\\ \text{Rec}=\frac{\text{TP}}{\text{TP}+\text{FN}}. \end{array}$$

First, this work analyzes the training process of MSRAFNET, and the analysis objects are training loss, training precision, and training recall. The changes of these three are demonstrated in Table 2.

As demonstrated in the data in the table, with the increase of network training iterations, the network loss shows a downward trend, and the network precision and recall rate show an upward trend. When the training iteration reaches 50 epochs, all three no longer change significantly, which indicates that network has tended to converge.

To verify the reliability of MSRAFNET designed in this work to evaluate the teaching quality of guzheng majors in colleges under big data, this work compares it with other methods, and the results are demonstrated in Figure 5.

The methods compared in this work include SVM, BP, DBN, CNN, and ResNet. Compared with these methods, MSRAFNET can achieve the highest precision and recall. Compared with other methods, MSRAFNET can achieve different degrees of improvement.

MSRAFNET uses a multiscale feature strategy. To verify the superiority of this strategy, the performances of single-scale features and multiscale features are compared, respectively. The comparison data is demonstrated in Figure 6.

Compared with single-scale features, after using multiscale features, MSRAFNET achieves 2.3% and 1.8% in precision and recall indicators, respectively, which confirms the superiority of multiscale features.

MSRAFNET uses a mixed attention mechanism. To verify the superiority of this strategy, the performances of not using mixed attention and using mixed attention are compared, respectively. The comparison data is demonstrated in Figure 7.

Compared with not using mixed attention, after using mixed attention, MSRAFNET achieves 1.5% and 1.1% in precision and recall indicators, respectively, which confirms the superiority of mixed attention.

MSRAFNET uses a transition layer. To verify the superiority of this strategy, the performances of not using transition layer and using transition layer are compared, respectively. The comparison data is demonstrated in Table 3.

Compared with not using transition layer, after using transition layer, MSRAFNET achieves 1.3% and 1.0% in precision and recall indicators, respectively, which confirms the superiority of transition layer.

MSRAFNET uses a global average pooling. To verify the superiority of this strategy, the performances of not using GAP and using GAP are compared, respectively. The comparison data is demonstrated in Figure 8.

Compared with not using GAP, after using GAP, MSRAFNET achieves 1.4% and 1.5% in precision and recall indicators, respectively, which confirms the superiority of GAP.

MSRAFNET uses a Dropout strategy. To verify the superiority of this strategy, the performances of not using Dropout and using Dropout are compared, respectively. The comparison data is demonstrated in Table 4.

Compared with not using Dropout, after using Dropout, MSRAFNET achieves 1.5% and 1.3% in precision and recall indicators, respectively, which confirms the superiority of Dropout.

### 4.2. Evaluation on Optimization Paths of Guzheng Professional Education

This work proposes some optimization paths for issues faced by the professional education of guzheng in colleges under big data. To verify feasibility of these optimization measures, this work compares the teaching quality of Guzheng before and after using these optimization measures. The compared indicators are the same as those in Table 1, and the comparison data is demonstrated in Figure 9.

Compared with before using the optimization measures, after using the proposed optimization path, every index of the quality of guzheng education in colleges can get a certain degree of score improvement. This verifies correctness as well as superiority of the optimized path proposed in this work.

## 5. Conclusion

With development for national economy, people's material and cultural level are further improved. Under such an environment, national culture has been paid more and more attention by people. Guzheng is a traditional Chinese national musical instrument, which combines musical beauty and beautiful shape. Guzheng provides people with a deep audio-visual experience and is a significant content in current college music teaching, which can cultivate students' sense of rhythm and aesthetic ability. However, there are still various issues in the current guzheng teaching in colleges, which affect good development of guzheng teaching. As the number of students has been growing steadily, on the one hand, the traditional teaching makes it difficult to maintain enthusiasm for learning the guzheng and cannot meet the needs of students to show their personal talents. The knowledge and skills learned do not have the opportunity to practice and make substantial progress through communication. This work studies the guzheng professional education in colleges under big data. First, this work aims at existing outstanding issues of guzheng teaching in colleges and studies the challenges and optimization paths of guzheng professional education in colleges under big data. Second, this work proposes a MSRAFNET to evaluate the teaching quality of guzheng majors in colleges under big data. The feature extraction of the network model is mainly completed by the residual module, which is composed of several multiscale residual learning units. Adding an attention mechanism to the multiscale residual learning unit can enhance the feature extraction of key information by the network and reduce the interference of redundant information, which is more conducive to the learning of data features. It adopts the design of GAP and Dropout to reduce spatial parameters in network training, and the effect of antioverfitting is better. Third, this work systematically evaluates the optimization path of Guzheng education and MSRAFNET, and the systematic experiments verify the feasibility and superiority of the designed method.

## Figures and Tables

**Figure 1:** MSRAFNET framework.

**Figure 2:** Multiscale residual learning unit.

**Figure 3:** Multiscale attention residual learning unit.

**Figure 4:** Transition layer structure.

**Figure 5:** Comparison with other methods.

**Figure 6:** Comparison of single-scale feature and multiscale feature.

**Figure 7:** Comparison of using mixed attention and not using mixed attention.

**Figure 8:** Comparison of using GAP and not using GAP.

**Figure 9:** Evaluation on optimization paths of guzheng professional education.

**Table 1:** The data feature contained in each sample.

Feature	Index
Teaching objective	X1
Teaching content	X2
Teaching attitude	X3
Teaching method	X4
Teaching atmosphere	X5
Playing skill	X6
Humanistic literacy	X7
Practical ability	X8

**Table 2:** MSRAFNET training analysis.

Epoch	10	20	30	40	50	60	70	80	90	100
Loss	3.41	1.53	0.72	0.52	0.41	0.41	0.39	0.39	0.40	0.39
Precision	83.2	89.1	94.1	96.2	98.3	98.2	98.3	98.1	98.2	98.2
Recall	75.3	81.5	92.2	93.6	95.2	95.3	95.3	95.1	95.2	95.1

**Table 3:** Comparison of using transition layer and not using transition layer.

Method	Precision	Recall
Not using transition layer	94.3	92.2
Using transition layer	95.6	93.2

**Table 4:** Comparison of using Dropout and not using Dropout.

Method	Precision	Recall
Not using Dropout	94.1	91.9
Using Dropout	95.6	93.2

## Data Availability

The datasets used during this study can be obtained from the corresponding author upon reasonable request.
